The article "Synergistic Preparation of Sludge Carbon from Oily Sludge and Walnut Shells" was published in 2022. Journal: Int J Anal Chem.

# Synergistic Preparation of Sludge Carbon from Oily Sludge and Walnut Shells

**DOI:** 10.1155/2022/6734039

**Published:** 2022-08-18

**Authors:** Chao Tang, Jiaojiao Guan

**Affiliations:** ^1^Chongqing Water Resources and Electric Engineering College, Chongqing 402160, China; ^2^State Key Laboratory of Petroleum and Pollution Control, Beijing 102206, China

## Abstract

The preparation process of synergistic preparation of sludge carbon by oily sludge and walnut shells are divided into two stages: carbonization preparation of a carbon precursor and activation preparation of sludge carbon. The preparation conditions of the carbon precursor are 2.5:1 mass ratio of oily sludge and walnut shells, carbonization temperature is 450°C, and time is 2 h. There are some pores on the surface of the prepared carbon precursor, the heavy metal content of leachate does not exceed the standard, and the use process will not cause heavy metal pollution. Intensive research is carried out on factors affecting the preparation of sludge carbon by activation of the carbon precursor by the orthogonal experiment and single-factor experiment. The optimal activation conditions are determined by using ZnCl_2_ as an activator, mass ratio of the carbon precursor to ZnCl_2_ is 1:4, activation temperature is 800°C, heating rate is 15°C/min, and activation holding time is 1 h. The surface of sludge carbon is distributed with many pores, several layers of small pores can be seen deeply in the large holes, and pore size distribution is dominated by micropores and mesopores. BET Specific surface area, pore volume, average pore, and iodine value are 1772.69 m^2^/g, 1.98 cm^3^/g, 1.64 nm, and 1011.65 mg/g, respectively, which surpasses commercially available activated carbon comprehensively.

## 1. Introduction

Oily sludge is the most important oily solid waste in the process of oil and gas field development. Because of its great harm to the ecological environment, China identified it as hazardous solid waste in the “National Catalogue of Hazardous Wastes” in 1998, and it continues to be retained in the newly revised list in 2021 [1–3]. China's new environmental protection law also further lowers the threshold for sentencing and convicting environmental pollution accidents, which reflect China's high standards and strict requirements for the treatment and disposal of hazardous solid waste in oil and gas fields on oily sludge [4]. Walnut shells are typical agricultural wastes, and China's walnut planting volume ranks top in the world. A large number of walnut shells produced after deep processing every year are mostly disposed in the form of fuel and filter material, and the comprehensive utilization of walnut shells has not been deeply developed [5].

The article "Synergistic Preparation of Sludge Carbon from Oily Sludge and Walnut Shells" was published in 2022. Journal: Int J Anal Chem.

Oily sludge has the potential to prepare activated carbon, but its viscous texture and poor dispersibility are not conducive to large-scale production. The preparation of activated carbon from agricultural and forestry wastes has been widely carried out [6–8], and there are also some reports on the preparation of activated carbon by mixing these two different types of materials. Wang et al. mixed sludge with rice husks to prepare activated carbon with abundant micropores and mesopores, and the specific surface area is 2575 m^2^/g, which is much higher than that of activated carbon prepared from a single raw material under the same preparation method [9]. Meng et al. mixed coal tar pitch and sawdust and prepared activated carbon with porous structure through chemical activation, and the specific surface area is 2224 m^2^/g [10]. However, the research on the preparation of activated carbon by mixed pyrolysis of two substances is still in its infancy, with few practical applications.

In this paper, sludge carbon was prepared synergistically by oily sludge and walnut shells. It not only deals with hazardous waste oily sludge which plague green development of oil and gas fields and agricultural waste walnut shells but also realizes resource utilization of two kinds of wastes, which fully reflected the concept of “green economy and circular development.”

## 2. Experimental

### 2.1. Materials

Oily sludge was from LiaoHe Oilfield, which was black and viscous. The water content, oil content, and residue content were 82.2%, 9.2%, and 8.6%, respectively. Walnut shells was from Shijiazhuang Baori Environmental Technology Co., Ltd. It was dried in an oven at 105°C for 24 h and then pulverized and ground to 50 mesh. The analysis results of elements and contents were C: 44.12%, H: 6.28%, O: 44.82%, N: 0.67%, and S: 0.18%.

### 2.2. Preparation Method of Sludge Carbon

Oily sludge and walnut shell powder were mixed evenly according to a certain mass ratio and placed into a tube furnace for carbonization. The carbonization process was protected by nitrogen. After carbonization was completed and cooled, the massive carbonized material was taken out and ground to 100 mesh, which was the carbon precursor. Then, the carbon precursor and activator were fully mixed in a certain proportion and activated ina tube furnace by nitrogen atmosphere. After activation was completed, the material was washed with dilute hydrochloric acid until the acid soluble was fully dissolved, and then washed with deionized water to neutral, drying to obtain sludge carbon. During the experiment, the heating rate of the tube furnace was 15°C/min, and the nitrogen flow rate was 100 mL/min.

The article "Synergistic Preparation of Sludge Carbon from Oily Sludge and Walnut Shells" was published in 2022. Journal: Int J Anal Chem.

### 2.3. Characterization of Products

Determination of the iodine value was based on the standard of GB/T 12496.8-2015. The elemental analysis was adopted by Quantax 200XFlash5000-10 EDS. Analysis of surface properties and SEM were determined by N_2_ adsorption ASAP and the Quanta250 tungsten filament scanning electron microscope, respectively. Heavy metal pollutants were analyzed by iCAP RQ ICP-MS.

## 3. Results and Discussion

### 3.1. Preparation of the Carbon Precursor

The preparation of sludge carbon was divided into two stages: carbonization and activation. The purpose of carbonization was to prepare the carbon precursor. Through carbonization, the organic components in the mixture were thermally decomposed to form the precursor with certain mechanical strength and pore structure [11]. In this study, the preparation conditions of the carbon precursor were as follows: mass ratio of oily sludge to walnut shell was 2.5:1, carbonization temperature was 450°C, and carbonization time was 2 h. After the reaction was completed, the lumpy carbides were ground to 100 meshes, which was the carbon precursor.

The iodine value of the carbon precursor was 304.77 mg/g, which indicated that the carbon precursor had initial porosity and partially adsorption capacity.  Table 1 showed the element composition of the carbon precursor indicating that the carbon precursor were mainly composed of C, Na, Al, Ca, and other metal oxide salts and silicon oxides.  Table 2 showed the composition and content of heavy metals in the carbon precursor indicating that the heavy metal content in the leaching solution of the carbon precursor was less than regulation values of “Identification Standards for Hazardous Waste Identification for Extraction Toxicity” and the first-order of “Integrated Wastewater Discharge Standard” in China, which displayed that sludge carbon further activated by the carbon precursor and prepared sludge carbon will not cause heavy metal pollution in the subsequent use process.

### 3.2. Preferred Activators

The first step in preparation of sludge carbon by carbon precursor activation was to select a suitable activator. A good activator has strong “pore-making” and “etching” ability, which can effectively expand the old pores and react to form new pores, which also has a catalytic effect, forming good pore structure and pore size distribution [12]. In this study, three commonly used activators (ZnCl_2_, AlCl_3_, and KOH) were selected [13, 14], and the effects of different activators on the adsorption performance of prepared sludge carbon were discussed.

Table 3 showed the iodine value of prepared sludge carbons when the activation temperature was 800°C, the heating rate was 15°C/min, the activation holding time was 1 h, and the mass ratio of carbon precursor to activator was 1:2 indicating that ZnCl_2_ had the best activation effect, and the prepared sludge carbon had the highest iodine value. Since ZnCl_2_ can reacted with the carbon in carbon precursor to form new pores, at the same time expanded the initial pores and pore channels in the carbon precursor to form a good pore structure [15].

The article "Synergistic Preparation of Sludge Carbon from Oily Sludge and Walnut Shells" was published in 2022. Journal: Int J Anal Chem.

### 3.3. Orthogonal Experimental of Sludge Carbon Preparation

There are four main factors affecting the activation stage of the carbon precursor to prepare sludge carbon, which are the mass ratios of the carbon precursor to ZnCl_2_, activation temperature, heating rate, and activation holding time. In this study, an orthogonal experiment of 3 levels and 4 factors L9 (3^4^) was designed, and the adsorption performance of prepared sludge carbon was characterized by the iodine value in order to obtain the most suitable activation conditions.

Tables 4 and 5 were the factor level tables and results of the orthogonal experiment, respectively, indicating that activation temperature was the most influential factor in the activation stage of preparation of sludge carbon, followed by activation holding time and mass ratio of the carbon precursor to ZnCl_2_, and the last was the heating rate. The calculated mean value displayed that the optimal levels of four influencing factors were *A*3, *B*2, *C*3, and *D*1, respectively. Therefore, the optimal activation conditions for preparation of sludge carbon were that the mass ratio of the carbon precursor to ZnCl_2_ was 1:4, the activation temperature was 800°C, the heating rate was 15°C/min, and the activation holding time was 1 h.

### 3.4. Single Factor Experimental of Sludge Carbon Preparation

In order to further explore the influence of three main factors: activation temperature, activation holding time, and mass ratio of the carbon precursor to ZnCl_2_ on the adsorption performance of sludge carbon, single-factor analysis was carried out respectively.

#### 3.4.1. Influence of the Mass Ratio of the Carbon Precursor to ZnCl_2_

Figure 1 showed the change of the iodine value of sludge carbon under different mass ratios of the carbon precursor to ZnCl_2_ when the activation temperature was 800°C, the heating rate was 15°C/min, and the activation holding time was 1 h, indicating that with the increase in the amount of activator ZnCl_2_, the iodine value of sludge carbon had also risen. This is because the activator ZnCl_2_ continuously squeezed between the carbon layers, and the activation reaction gradually expanded from the outer surface to the inside of particles, which promoted the development of pores of the carbon precursor and formed a large number of micropores at high temperature. When the mass ratio of the carbon precursor to ZnCl_2_ was 1:4, the iodine value of sludge carbon reached the maximum, and then the iodine value of activated carbon showed a downward trend with the continuous increase of ZnCl_2_. Due to the effect of pore structure, the pores of the carbon precursor are overactivated, the pore size gradually becomes larger [16], and the proportion of macropores increased.

The article "Synergistic Preparation of Sludge Carbon from Oily Sludge and Walnut Shells" was published in 2022. Journal: Int J Anal Chem.

#### 3.4.2. Influence of the Activation Temperature

Figure 2 showed the change of the iodine value of sludge carbon under different activation temperatures when the mass ratio of the carbon precursor to ZnCl_2_ was 1:4, the heating rate was 15°C/min, and the activation holding time was 1 h, which displayed that when the activation temperature was low, the iodine value of sludge carbon was small because the effective pore structure cannot be formed when the reaction was insufficient. When the activation temperature was too high, which would lead to the collapse of the micropore wall formed by activation in sludge carbon, and the proportion of macropores would increase, resulting in a decrease in the iodine value. Therefore, the suitable activation temperature was 800°C.

#### 3.4.3. Influence of the Activation Holding Time

Figure 3 showed the change of the iodine value of sludge carbon under activation holding time when the mass ratio of the carbon precursor to ZnCl_2_ was 1:4, the activation temperature was 800°C, and the heating rate was 15°C/min, which indicated that the optimal activation holding time for preparation of sludge carbon was 1 h. When activation holding time was too short, the iodine value was low because the precursor was not fully activated, the pore expansion was insufficient, and sufficient microporous structures cannot be formed. After activation holding time exceeded 1 h, the precursor was overactivated, which led to collapse of the pore structure and decrease of the iodine value.

### 3.5. Characterization of Sludge Carbon

Sludge carbon was obtained and characterized under the best preparation conditions (mass ratio of the carbon precursor to ZnCl_2_ was 1:4, activation temperature was 800°C, heating rate was 15°C/min, and activation holding time was 1 h), and the comparative study with commercially available activated carbon was performed.  Figure 4 was the SEM images of the carbon precursor, sludge carbon, and activated carbon, respectively, indicating that carbon precursor particles were tightly packed, and some pores and cracks of different sizes can be seen, but these pores and cracks were occupied and blocked by various small particles, and the pore structure was not obvious. Sludge carbon had an obvious structure with numerous pores distributed on the surface, and several layers of small pores can be seen in the depth of the large pores, which displayed that the activation process greatly expanded the pore structure of sludge carbon. The surface of activated carbon was smooth, and the pore structure was dominated by micropores with uniform distribution relatively.  Figure 5 showed the pore distribution of sludge carbon indicating that the pore-distribution of sludge carbon was relatively concentrated, mainly micropores and mesopores, and the proportion of micropores was high, especially a pore diameter of 1 nm. Surface properties and the iodine value of sludge carbon and activated carbon were analyzed. The results in Table 6 displayed that sludge carbon surpassed activated carbon in terms of the specific surface area, pore structure values, and iodine value. The specific surface area value was even more than double that of activated carbon. This showed that sludge carbon had strong performance, and the effect will be definitely stronger than that of activated carbon when applied to the field of activated carbon. Since one of the raw materials for preparation of sludge carbon was oily sludge, it may have strong lipophilic properties and special effects when applied to treatment of oily wastewater or organic wastewater [17], and further popularization and use need to be further studied.

The article "Synergistic Preparation of Sludge Carbon from Oily Sludge and Walnut Shells" was published in 2022. Journal: Int J Anal Chem.

## 4. Conclusions

Sludge carbon was prepared synergistically by combining carbonization and activation with oily sludge and walnut shells as raw materials. The conditions for carbonization to the prepared carbon precursor were that the mass ratio of oily sludge to walnut shells was 2.5:1, the carbonization temperature was 450°C, and the carbonization time was 2 h. The conditions for activation of prepared sludge were as follows: ZnCl_2_ was used as an activator, the mass ratio of the carbon precursor to ZnCl_2_ was 1:4, the activation temperature was 800°C, the heating rate was 15°C/min, and the activation holding time was 1 h. The prepared sludge carbon had excellent pore characteristics, and the pore size distribution was dominated by micropores and mesopores. The BET specific surface area, pore volume, average pore size, and iodine value all exceed those of commercially available activated carbon, reaching 1772.69 m^2^/g, 1.98 cm^3^/g, 1.64 nm, and 1011.65 mg/g, respectively.

## Figures and Tables

**Figure 1:** The influence of the mass ratio of the carbon precursor to ZnCl_2_ on the iodine value of sludge carbon.

The article "Synergistic Preparation of Sludge Carbon from Oily Sludge and Walnut Shells" was published in 2022. Journal: Int J Anal Chem.

**Figure 2:** The influence of the activation temperature on the iodine value of sludge carbon.

**Figure 3:** The influence of the activation holding time on the iodine value of sludge carbon.

**Figure 4:** SEM of (a) the carbon precursor, (b) sludge carbon, and (c) activated carbon.

**Figure 5:** The pore-distribution curve of sludge carbon.

**Table 1:** Mass fractions of elements in the carbon precursor.

Sample	Elemental composition and their mass fractions (%)						
	C	O	Na	Al	Si	S	Ca
Carbon precursor	48.26	27.71	1.04	5.96	5.47	0.98	2.37

**Table 2:** Extraction toxicity of heavy metals in the carbon precursor (mg/L).

Sample	Cr	Hg	Ni	Cu	Zn	Cd	Pb	As
Carbon precursor	0.028	0.006	0.260	0.710	0.341	0.017	0.024	0.014
*A*	15	0.1	3	100	100	1	5	5
*B*	1.5	0.05	1	0.5	2.0	0.1	1.0	0.5

*A*: regulation values of “identification standards for hazardous wastes-identification for extraction Toxicity.” *B*: first-order of “integrated wastewater discharge standard.”

**Table 3:** Preferred activators.

Activators	Iodine value (mg/g)
ZnCl_2_	988.32
AlCl_3_	657.14
KOH	948.43

**Table 4:** Orthogonal factor level table L9 (3^4^).

Level	Factor *A*	Factor *B*	Factor *C*	Factor *D*
	Mass ratio of the carbon precursor to ZnCl_2_	Activation temperature (°C)	Heating rate (°C/min)	Activation holding time (h)
1	1:1	650	5	1
2	1:2	800	10	2
3	1:4	950	15	3

**Table 5:** Optimization of activation condition orthogonal analysis results.

Number	Factor and level				Iodine value (mg/g)
	*A*	*B*	*C*	*D*	
1	1	1	1	1	598.61
2	1	2	2	2	676.51
3	1	3	3	3	629.89
4	2	1	2	3	570.12
5	2	2	3	1	988.32
6	2	3	1	2	708.07
7	3	1	3	2	576.81
8	3	2	1	3	770.27
9	3	3	2	1	939.76

*k*1	635.003	581.847	692.317	842.230	
*k*2	755.503	811.700	728.797	653.797	
*k*3	762.280	759.240	731.673	656.760	
*R*	127.277	229.853	39.356	188.433	

Order	*B* > *D* > *A* > *C*				

Optimal level	*A*3	*B*2	*C*3	*D*1	

Optimized combination	*A*3 *B*2 *C*3 *D*1				

**Table 6:** Surface characteristics and the iodine value of sludge carbon and activated carbon.

Sample	BET specific surface area (m^2^/g)	Pore volume (cm^3^/g)	Average pore size (nm)	Micropore ratio (%)	Iodine value (mg/g)
Sludge carbon	1772.69	1.98	1.69	35.3	1011.65
Activated carbon	883.21	0.46	2.48	28.9	716.31

## Data Availability

The table data, figure data, and other related data used to support the findings of this study are included within the article.
